The article "Role of Estrogen Receptor-Positive/Negative Ratios in Regulating Breast Cancer" was published in 2022. Journal: Evid Based Complement Alternat Med.

# Role of Estrogen Receptor-Positive/Negative Ratios in Regulating Breast Cancer

**DOI:** 10.1155/2022/7833389

**Published:** 2022-09-08

**Authors:** Yanchu Li, Hengli Zhang, Tingting Jiang, Ping Li

**Affiliations:** ^1^Head & Neck Oncology Ward, Cancer Center, West China Hospital of Sichuan University, Chengdu, Sichuan, China; ^2^Department of Oncology, Cancer Prevention and Treatment Institute of Chengdu, Chengdu Fifth People's Hospital (The Second Clinical Medical College, Affiliated Fifth People's Hospital of Chengdu University of Traditional Chinese Medicine), Chengdu, China

## Abstract

The alpha estrogen receptor (ER*α*) contributes to breast cancer progression and recent guidelines define ER positivity as ≥1% stained cells, and a few tumor tissues show no ER*α* expression at all or are at 100%. Although ER and aromatase inhibitors are widely used to treat hormone receptor-positive (HR+) breast cancer, their effect on tumor activity at different ER*α* levels remains unclear. Therefore, we investigated the role of ER*α*+/ER*α*− ratios in determining the ER*α* level. We used ER*α* stably transfected and wild-type MDA-MB-231 cells (MDA-MB-231^Trans−ER^ and MDA-MB-231^WT^, respectively) as represented ER+ and ER− cells, respectively, and MCF-7 cells were the positive control. MDA-MB-231^Trans−ER^ and MDA-MB-231^WT^ cells were mixed and cocultured at a ratio of 0%, 20%, 40%, 70%, and 100%. Migration and invasion functions at different cell ratios were evaluated in vitro using the Transwell and scratch test. In a xenograft mouse model, the polarization of the tumor-associated (M2) macrophage and the expression of breast cancer gene 1 (BRCA1), human epidermal growth factor receptor 2 (HER2), vascular endothelial growth factor (VEGF), and tumor necrosis factor (TNF)-*α* were measured. The results showed that the cell invasion and migration were significantly higher at 40% and 70% than they were at other ratios. Additionally, in vivo, the 70% ER*α*+/ER*α*-ratio was a critical indicator of cell activity and cytokine expression. The highest M2 level and expression of VEGR, TNF-*α*, BRCA1, and HER2 were shown at a ratio of 70%. Moreover, the effects of ER*α* were not linear in breast cancer, indicating that the ER*α* status requires continuous monitoring during long-term endocrine treatment. These results indicate that during HR+ breast cancer treatment, the ER*α*+/ER*α*− ratio may be a useful predictor and should be evaluated further.

## 1. Introduction

Worldwide, cancer is the second leading cause of death and breast cancer is the most common cancer in women [1]. Most breast cancers show an overexpression of the estrogen receptor (ER). Antiestrogen therapy with agents such as tamoxifen (TAM) and aromatase inhibitors is the cornerstone of systemic breast cancer therapy, which has significantly improved the survival of women with hormone receptor-positive (HR) breast cancers [2–4]. Because the ER status is essential for patient management, it is important to ensure it is assessed accurately [5]. Estrogens exert their biological effects through binding to ER*α* and ER*β* [6].

The article "Role of Estrogen Receptor-Positive/Negative Ratios in Regulating Breast Cancer" was published in 2022. Journal: Evid Based Complement Alternat Med.

Studies have reported that approximately 60–70% of breast cancer patients express ER, which is implicated in the progression of breast cancer. Tumor progression, endocrine therapy, and prognosis are closely related to the expression level of ER. The updated American Society of Clinical Oncology/College of American Pathologists (ASCO/CAP) guidelines classify tumors with ER expression 1–10%, >10%, and <1% as ER-low+, ER+, and ER− breast tumors, respectively. Paakkola et al. [7] reported that ER-low+ breast cancer had a more similar outcome to that of ER− than to ER+ breast cancer in disease-free survival (DFS) and overall survival (OS) and discussed the prognosis based on ER status.

The prognosis of ER*α*+ breast cancer is better than that of ER*α*−, and ER expression is also related to bone and visceral metastasis [8]. Interestingly, ER*α*+ patients primarily show metastasis to the bone, skin, or soft tissue, whereas that of ER*α*− patients is more common in the lungs, liver, and brain. Singhakowinta [8] showed that although treating reexpressed ER cell lines with estradiol reduced aggressiveness, applying TAM to ER+ cells may increase the risk of lung metastasis in mice [9]. Moreover, results of recent studies indicate that transfecting fluorescence-tagged MDA-MB-435 (MDA-MB-435-FL) and MDA-MB-231 ER+ cells with the ER prevented bone metastasis [10]. However, the effect on tumor activity at the different ER*α* levels was not considered.

Currently, research on endocrine therapy in breast cancer is gradually advancing, but the relationship between the balance of ER*α* expression and the best benefit for breast cancer patients is still not clear. Thus, although TAM and aromatase inhibitors are effective and have been widely used to treat ER+ breast cancer, determining the appropriate level of ER*α* suppression and exploring the balance of the ER expression in the tumor microenvironment is required. Previous studies have reported that the function of ER+ is not always consistent and linear. Thus, this study established a cell line and xenograft model with different ER*α*+/ER*α*− ratios to identify the least favorable and lethal ratio and its underlying mechanism.

## 2. Methods

### 2.1. Cell Lines and Culture

MDA-MB-231^WT^ and MDA-MB-231^Trans−ER^ cell lines were used as representative ER− and infectant ER+ human breast cancer cells, respectively, as the experimental groups and MCF-7 cells were the ER+ control group. Cells were cultured in Dulbecco's modified Eagle's medium (DMEM, Thermo Scientific HyClone, USA) containing 10% fetal bovine serum (FBS) and 1% penicillin and streptomycin, at 37°C in an atmosphere of 5% CO_2_.

The article "Role of Estrogen Receptor-Positive/Negative Ratios in Regulating Breast Cancer" was published in 2022. Journal: Evid Based Complement Alternat Med.

### 2.2. ER*α* Stable Transfection

MDA-MB-231^WT^ cells were seeded (1 × 10^5^ cells/well) in 24-well plates and were stably transfected with the ER*α* expression plasmid (pEGFP-C1-ERa) using Lipofectamine™ 2000 (Invitrogen, USA). Then, 500 *μ*L Opti-MEM ® I low serum medium (DNA : Lipofectamine 2000 = 1 : 3, containing 2 *μ*L Lipofectamine and 0.8 *μ*g plasmid DNA) was added and the mixture was incubated at room temperature (26°C) for 20 min to form the complex and then cultured in a 37°C CO_2_ incubator for 48 h. Then, a G418-containing medium (800 *μ*g/mL) was added to the screen, and breast cancer cells stably expressing plasmid enhanced green fluorescence protein (PEGFP)-C1-ER*α* were obtained and designated as MDA-MB-231^Tran−ER^.

### 2.3. Cocultured Cells at Different MDA-MB-231^Trans−ER^/MDA-MB-231WT Ratios

MDA-MB-231^WT^ and MDA-MB-231^Trans−ER^ cells were mixed and cocultured at 100%, 70%, 40%, 20%, and 0% ratios as the experimental group (ER*α*+/ER*α*−) and the MCF-7 cell line was the control group. ER protein from each group was analyzed using immunofluorescence staining.

### 2.4. 3-(4,5-Dimethylthiazol-2-yl)-2,5-diphenyltetrazolium Bromide Assay of Cell Viability

Cell viability was assessed using the 3-(4,5-dimethylthiazol-2-yl)-2,5-diphenyltetrazolium bromide (MTT) assay (Sigma-Aldrich, USA). MDA-MB-231^WT^, MDA-MB-231^Trans−ER^, and MCF-7 cells were seeded (1 × 10^3^ cells/well) in 96-well plates. After 24, 48, 72, 96, 120, and 144 h incubation, 20 *μ*L 5 mg/mL MTT solution was added to each well, and the plate was further incubated at 37°C for 4 h. Then, the medium was aspirated and 200 *μ*L dimethyl sulfoxide (DMSO) was added to each well. After the formazan crystals had dissolved, the absorbance was determined spectrophotometrically at 492 nm using a BioTek *μ*Quant™ reader (BioTek, USA).

### 2.5. Cell Scratch Assay of Migration Ability

Cell migration ability was quantitated using the cell scratch assay. Briefly, MDA-MB-231^Trans−ER^ and MDA-MB-231^/WT^ cells (2 × 10^4^ cells) at 0%, 20%, 40%, 70%, and 100% ER*α*+/ER*α*−ratios were placed into each well of a six-well plate ensuring that each well was coated with cells. Then, a 1 mL pipette tip was used to scratch cells at the bottom of the well, and the plates were washed with phosphate-buffered saline (PBS) three times to remove the displaced scratched cells. Cells were cultured in an incubator at 37°C in an atmosphere of 5% CO_2_. Images of the samples were captured at 24 h and 48 h using the Eclipse TS100 microscope (Nikon, Japan), and this procedure was repeated three times.

The article "Role of Estrogen Receptor-Positive/Negative Ratios in Regulating Breast Cancer" was published in 2022. Journal: Evid Based Complement Alternat Med.

### 2.6. Transwell Assay of Cell Migration

Transwell cell culture inserts were coated with appropriately diluted Matrigel and 2 mL of the cell suspension from each group was added to the Transwell chamber, which was then immersed into a 24-well plate. After incubating at 37°C in an atmosphere of 5% CO_2_ for 48 h, the Transwell chamber was washed gently with PBS, the cells were fixed with 4% paraformaldehyde, and then the cells on the membrane surface of the upper chamber side were wiped with a cotton swab, retaining the cells on the surface of the lower chamber side. The number of invading cells was counted under an Eclipse TS100 microscope.

### 2.7. Xenograft Mouse Breast Cancer Model

Female-specific, pathogen-free, (SPF)-Balb/*c* mice weighing 21 ± 1.2 g were brought from the DaShuo Company (Chengdu, China). The animal study was approved by the Institutional Animal Care and Use Committee. MDA-MB-231 cells at 0%, 20%, 40%, 70%, and 100% ER*α*+/ER*α*− ratios and MCF-7 cells were transplanted into the right dorsal side of each mouse at 1 × 10^6^ cells/mouse for each cell line. Then, 25 MDA-MB-231 tumor-bearing mice were divided into five groups (*n* = 5 each) and the MCF-7 cell tumor-bearing mice served as the control (*n* = 5).

### 2.8. Reverse Transcription-Polymerase Chain Reaction (RT-PCR)

RNA was extracted from cell and tissue samples from the MDA-MB-231^Trans−ER^/MDA-MB-231^WT^ group with different ratios. Specific primers were used to amplify the ER*α*, human epidermal growth factor receptor 2 (HER2), and progesterone receptor (PR) from the cDNA. Briefly, 1 *μ*g of the total RNA was reverse transcribed in a total reaction volume of 20 *μ*L using 1 *μ*L each of iScript reverse transcriptase and 5 × iScript reaction mix. The resulting cDNA was then diluted to 20 *μ*L with RNase-free water (H_2_O) and each RT-PCR sample consisted of 1 *μ*L diluted RT product, 1 × SYBR Premix Ex Taq™ II 10 *μ*L, and 0.4 *μ*mol each of the forward and reverse primers. Reactions were conducted by using an LC480 system (Roche, USA) for 40 cycles (95°C for 5 s and 60°C for 30 s) after an initial 30 s incubation at 95°C.

### 2.9. Immunohistochemistry (IHC) and Immunofluorescence (IF) Assay

Tumor tissues were fixed in 10% buffered formalin, embedded in paraffin, and cut into sections, which were then dewaxed with dimethyl-benzene and hydrated with different decreasing concentrations of ethanol (100%, 95%, 85%, 70%, and 50%). The endogenous peroxidase activity was blocked by incubating the sections in a 3% hydrogen peroxide (H_2_O_2_) solution, followed by unmasking of the antigenic epitope with citrate buffer. Then, the sections were blocked by incubation in blocking buffer, followed by incubation with primary antibodies against vascular endothelial growth factor (VEGF), TNF-*α*, and ER (IF) and the appropriate secondary antibody. Finally, 3,3′-diaminobenzidine (DAB, Beyotime, China) substrate solution was applied to the sections to develop the color of the antibody staining. Three pathological sections from each group were examined, and the highest expression or negative section of each group was selected. The selected images were acquired by using an Eclipse TS100 microscope, and the ImageJ software with immunohistochemistry (IHC) profiler plugin (1.53 K, National Institute of Health (NIH), USA) was used to quantify the TNF-*α* and VEGF expression levels.

The article "Role of Estrogen Receptor-Positive/Negative Ratios in Regulating Breast Cancer" was published in 2022. Journal: Evid Based Complement Alternat Med.

### 2.10. Western Blot Assay

The tumor tissues were lysed in lysis buffer and then centrifuged at 15,000 rpm for 15 min at 4°C. The protein concentration was determined using a bicinchoninic acid (BCA) kit (Beyotime, China). A total of 50 *μ*g of protein was separated using 8% sodium dodecyl sulfate-polyacrylamide gel electrophoresis (SDS-PAGE) and transferred onto a polyvinylidene fluoride (PVDF) membrane (Merck Millipore, USA). The membranes were blocked for 1 h at 26°C with 5% bovine serum albumin containing 0.1% Tween-20, incubated with the primary antibodies (breast cancer gene 1 (BRCA1) and HER2, Beyotime, China; 1 : 1000) overnight at 4°C. Then, the membranes were washed with Tris-Buffered Saline with Tween-20 (TBST) three times and incubated with the corresponding secondary antibody (1 : 5000) at 37°C for 2 h. The membranes were then washed again and the proteins were detected using an enhanced chemiluminescence assay kit (Beyotime, China), followed by image capturing using the BioRad XRS + imaging system (BioRad, USA).

### 2.11. Flow Cytometry Assay

Cells were separated from the different MDA-MB-231^Trans/WT^ ratio tumor tissue and exposed to F4/80-phycoerythrin (PE; MF48004-3) and Ly6C-fluorescein isothiocyanate (FITC; 553104) fluorescent antibodies (both from BD Biosciences, USA) for flow cytometry. Cells were stained with F4/80-PE and Ly6C-FITC for 1h in the dark at 4°C and the samples were examined using the fluorescence-activated cell sorting (FACS) Caliber system (BD, USA).

### 2.12. Statistical Analysis

Results are expressed as means, and the difference between means was assessed using Student's *t*-test with Prism GraphPad 8.0. A *P* value < 0.05 was considered a statistically significantly difference.

The article "Role of Estrogen Receptor-Positive/Negative Ratios in Regulating Breast Cancer" was published in 2022. Journal: Evid Based Complement Alternat Med.

## 3. Results

### 3.1. Identification of ER*α* Transfection

As illustrated in Figure 1(a), the MDA-MB-231^WT^ cells were successfully and stably transfected with pEGFP-C1-ER*α*, which emitted green fluorescence and were designated as MDA-MB-231^Trans−ER^. The Western blot analysis results showed that ER*α* was strongly expressed in the transfected MDA-MB-231^Trans−ER^, indicating that the pEGFP-C1-ER*α* plasmid induced strong ER*α* expression in the MDA-MB- 231^WT^ cells (Figure 1(b)). Next, to identify the biological function of the MDA-MB-231 ^Trans−ER^, its optical density (OD) as well as those of the MDA-MB-231^WT^ and MCF-7 cells were detected from day 1 to day 6 (Figure 1(c)). Transfection of MDA-MB-231^WT^ with ER*α* significantly inhibited cell proliferation (*P* < 0.05), indicating that ER*α* affected cell viability.

To detect the ER*α* cell and tumor tissue expression of different ER*α*+/ER*α*− ratio groups, immunofluorescence and RT-PCR were used (Figure 2). The results showed a gradual reduction in the expression of ER*α* protein, which was correlated with the ER*α*+/ER*α*− ratio in vitro (Figure 2(a)). However, the ER*α* gene expression in the tumor tissue gradually increased consistently with different ER*α*+/ER*α*−ratios (Figure 2(b)). The results revealed that the MDA-MB-231^Trans−ER^/MDA-MB-231^WT^ model group was successfully established.

### 3.2. ER*α*+/Er*α*− Ratios Contributed to Regulate Cell Invasion and Migration

To study the invading capacity of cells, the Transwell test was used. As shown in Figure 3(a), the number of invading breast cancer cells at different ER*α*+/ER*α*− ratios (100%, 70%, 40%, 20%, and 0%) was 249 ± 6, 404 ± 28, 430 ± 25, 401 ± 25, and 361 ± 20 cells, respectively. According to the results, the highest cellular invasion capacity was observed at 40% and 70% ER*α*+/ER*α*− ratio. Furthermore, we investigated the effects of ER*α*+/ER*α*− ratio on cell migration and Figure 3(b) shows that scratched closure areas were observed for 48 h at various ratios of 0%, 20%, 40%, 70%, and 100%. Compared to the migration rate of the MCF-7 control cells, the values were 25.7 ± 2.5%, 31.7 ± 2.5%, 34.3 ± 1.5%, 37.0 ± 2.0%, and 26.7 ± 2.5% in 24 h (*P* < 0.05) and 55.3 ± 1.5%, 69.7 ± 2.1%, 77.7 ± 3.5%, 83.7 ± 5.0%, and 45.0 ± 3.0% in 48 h (*P* < 0.05) for cells at ER*α*+/ER*α*− ratios of 0%, 20%, 40%, 70%, and 100%, respectively. Based on these results, the greatest cell migration occurred at 40% and 70% ER*α*+/ER*α*− ratios.

The results showed that cell invasion and migration were more significantly stable at 40% and 70% ER*α*+/ER*α*− ratios than they were at the other ratios, including 100% ER*α*+/ER*α*− ratio. Thus, these findings indicate that various ER*α*+/ER*α*− ratios might affect cell functions in breast cancer.

The article "Role of Estrogen Receptor-Positive/Negative Ratios in Regulating Breast Cancer" was published in 2022. Journal: Evid Based Complement Alternat Med.

### 3.3. ER*α*+/Er*α*− Ratios Were Influential in Tumor Cytokine Expression

To investigate the relationship of TNF-*α* and VEGF expression to tumor progression, the tumor microenvironment of different ER*α*+/ER*α*− ratio groups was immunohistochemically analyzed. As illustrated in Figure 4, TNF-*α* and VEGF showed a weakly positive (+) expression in the 100% ER*α*+/ER*α*− ratio group, but were both strongly positive (+++) in the 40% and 70% ER*α*+/ER*α*− ratio groups, Furthermore, both the TNF-*α* and VEGF expression was strongly positive (+++) and higher than the medium positive (++) level observed with 0% and 20% ER*α*+/ER*α*−ratio groups (*P* < 0.05). These results indicate that the 70% ER*α*+/ER**α**− ratio could be considered an approximate cutoff value for levels that affect tumor progression.

### 3.4. ER*α*+/Er*α*− Ratios Affected Tumor Microenvironment

To further investigate the effect of the ER*α*+/ER*α*− ratio on the breast cancer microenvironment, tumor-associated (M2) macrophage polarization, which is related to the negative immune environment, and BRCA1/HER2 protein expression that correlates to breast cancer proliferation were evaluated in the tumor microenvironment. The results of the flow cytometric assessment of the polarization rate of M2 macrophages (Figure 5(a)) showed that the percentage of F4/80+ and Ly-6C + cells, which represent M2 macrophages, was 4.9 ± 0.7%, 6.2 ± 0.6%, 7.2 ± 0.5%, 7.7 ± 0.5%, and 5.0 ± 0.6% for the 0%, 20%, 40%, 70%, and 100% ER*α*+/ER*α*− ratios groups, respectively. Furthermore, the 70% ER*α*+/ER*α*− ratio group showed a significant M2 macrophage increase (*P* < 0.05). Moreover, the analysis of BRCA1 and HER2 protein expression showed higher levels in the 40% and 70% ER*α*+/ER*α*− ratio groups than in the other groups, especially the 70% ER*α*+/ER*α*−ratio group (Figure 5(b)).

## 4. Discussion

The invasiveness and migration capacity of breast tumor cells are currently known to correlate with ER expression, and in this study, we confirmed that breast cancer treatment was the most effective with an essential balance of the ER*α*+/ER*α*− ratio status. In this pilot study, transfected MDA-MB-231^WT^ (ER−) and MDA-MB-231^Trans−ER^ (ER+) cells were used to determine the effect of cell biofunctions in breast cancer at different ER*α*+/ER*α*−ratios. At the 70% ER*α*+/ER*α*−ratio, MDA-MB-231^Trans−ER^ and MDA-MB-231^WT^ cell models showed the strongest cell invasion and migration in vitro as well as the highest M2 macrophage polarization and VEGR, TNF-*α*, BRCA1, and HER2 expression levels in the tumor microenvironment. These findings indicate that the degree of tumor malignancy was the highest at a specific ER*α* ratio of approximately 70%, rather than 100%.

The article "Role of Estrogen Receptor-Positive/Negative Ratios in Regulating Breast Cancer" was published in 2022. Journal: Evid Based Complement Alternat Med.

Breast cancer is the most frequent female endocrine-associated malignancy, and the main comprehensive treatments include surgery, radiotherapy, chemotherapy, endocrine therapy, and biological targeted therapy [4, 11, 12]. Although the ER includes ER*α*, ER*β*, and ER*γ* subtypes, the expression of ER*β* and ER*γ* is weak in breast cancer cells. Previous studies suggest that not only ER is the the most effective predictor of the response of patients with breast cancer to endocrine therapy but also the extranuclear function of ER cells plays an important role in cell proliferation, movement, and metastasis [13]. Thus, determining the site and status of breast tumor ER is vital to effectively and successfully treat patients and ultimately improve outcomes and survival rates [12]. The results of the National Cancer Database and the Surveillance, Epidemiology, and End Results (SEER) program indicate that while single ER + or PR + tumor subtypes indicate a worse prognosis than ER+/PR + tumors, ER−/PR + tumors exhibit a similar prognosis to that of the ER−/PR−subtype [14–16]. Furthermore, the ER and PR status may change during the development and treatment of breast cancer [17]. Moreover, previous studies have reported a U-shaped relationship between the expression of the ER*α* and the risk of bone and visceral metastasis of breast cancer, and the ER*α* target expression was shifted to the positive side. These observations indicate that the ER+/ER−ratio is correlated with the malignant bioactivity and the growth capacity of breast cancer. Therefore, the conversion among ER+/PR+, single ER+, and ER−/PR+ needs be clearly elucidated.

Previous studies have reported that the ER+ function was not always consistent and linear [8]. For instance, the risk of bone metastasis in ER+ patients is higher than that in ER-negative patients, whereas, in contrast, with bone metastasis, the risk of visceral metastasis in ER+ patients is lower than that in ER− patients [8]. Garcia et al. [9] and Bandyopadhyay et al. [10] reported that the ER effectively reduced cell invasion and bone metastasis. Moreover, because of the heterogeneity of tumors, the definition of ER positivity is ≥ 1% stained cells, and only a few tumors tissue show no ER expression or are at 100% [18]. Moreover, during tumor development, some tumor cells with positive and negative HRs could be switched [13, 19]. Experiments by Koibuchi et al. [20] in nude mice during this process confirmed that by suppressing estrogen levels in athymic mice, TAM reduced the expression of ER*α*. However, Noguchi et al. [21] recognized that TAM enhances the expression of ER*α* in human breast cancer. The data showed that women with ER+ primary tumors that changed to ER− had a significant 48% increased risk of death [19]. Previous studies have confirmed that for ER+ and PR+ patients, selective ER modulators (SERM) were effective at 60%–70% [22]. However, for ER− and PR− patients, the effective rate was approximately 10% and nearly 50% of ER*α*+ patients did not respond to TAM [22].

The article "Role of Estrogen Receptor-Positive/Negative Ratios in Regulating Breast Cancer" was published in 2022. Journal: Evid Based Complement Alternat Med.

In addition, Src-kinase, mitogen-activated protein kinase (MAPK), and phosphatidylinositol-3-kinase (PI3K) pathways are associated with the ER-extranuclear signaling by rapidly responding to cytosolic estradiol. Emerging evidence indicates that the ER participates in extranuclear signaling through the formation of a multiprotein complex called “signal some” [23]. Moreover, the endogenous acid and leucine-rich protein (PELP1) was proposed to mediate the intranuclear function of ER+ cells and the ER-Src-PELP1-ILK1 pathway shows potential as a novel therapeutic target for ER+ metastasis. BRCA1+ tumors are usually accompanied by ER− expression and P53 expression [24]. In the tumor microenvironment, TNF-*α* secreted by tumor-associated M2 macrophages could increase the expression of matrix metalloproteinases (MMPs) and VEGF through the Jun-c N-terminal kinase (JNK) and nuclear factor (NF)-kB pathways to increase their invasiveness [25, 26].

In addition, although ER is a predictor of breast cancer, the prognosis involves a dynamic variation rule and is affected by the biological balance of the tumor microenvironment. Our study demonstrated that the representative breast cancer cells, which were ER*α*+ or ER*α*−, interacted with each other. The long-term use of estrogen inhibitors alters the status and percentage of the ER*α*+/ER*α*− ratio of the tumor microenvironment. Furthermore, overuse of estrogen inhibitors may disrupt the equilibrium of the ER+/ER− ratio, causing unexpected adverse effects. Both high and negative ER*α* expression are risk factors for breast cancer. Therefore, it is not ideal to inhibit the expression of ER*α*+ cells or to increase that of ER*α*−. Furthermore, this study showed the effect of different ER*α*+/ER*α*− ratios on VEGF and TGF-*β* expression, which would guide the use of VEGFR or TGF-*β* inhibitors in the treatment of patients with breast cancer who have different ER*α*+/ER*α*− ratios. However, we did not record or examine the overall survival difference between patients with ER*α*+/ER*α*−^high^ and ER*α*+/ER*α*−^low^ statuses.

Furthermore, in the present study, although the M2 macrophage polarization and expression of VEGR, TNF-*α*, BRCA1, and HER2 showed differences among the different ER*α*+/ER*α*− ratio groups, the tumor size was not significantly different. In addition, cytokine release in the tumor microenvironment was more sensitive than tumor size growth, and the balance of the ER*α*+/ER*α*− ratio was associated with tumor cell invasion and proliferation, which provided a nonlinear hormone microenvironment for tumor growth. Thus, these phenomena further illustrate that the role and of the ER*α*+/ER*α*− ratio needs to be clearly recognized and appropriately modulated to fully understand the malignant biological behavior of breast cancer. Furthermore, the balance of the ER*α*+/ER*α*− ratio might be an independent treatment factor and could guide treatment decisions.

The article "Role of Estrogen Receptor-Positive/Negative Ratios in Regulating Breast Cancer" was published in 2022. Journal: Evid Based Complement Alternat Med.

## 5. Conclusions

Breast cancer cell biology did not exhibit a linear function according to the ER*α*+ level. Different ER*α*+/ER*α*− ratios correlated with different biofunctions. Consequently, the ER expression level requires constant monitoring during endocrine treatment, which could be related to hormone therapy time. The results of this study indicate a predictive role for the ER*α*+/ER*α*− ratio in ER+ breast cancer prevention.

## Figures and Tables

**Figure 1:** Confirmation of ER*α* transfection. (a) ER*α* stably transfected in MDA-MB-231 cell. pEGFP-C1-ER*α* expression was observed (green fluoresce) 48 h after transfection. (b) Western blot assay: ER*α* protein highly expressed in MDA-MB-231^Trans−ER^ cells. (c) MTT assay. Compared to the MDA-MB-231^WT^ cells, the proliferation ability of MDA-MB-231^Trans−ER^ cells was significantly inhibited (*P* < 0.05) and was similar to that of MCF-7 cells.

**Figure 2:** ER*α* expression (red) *in vitro* and *in vivo*. (a) *In vitro* evaluation of ER*α* expression in cocultured MDA-MB-231^Trans−ER^ (ER*α*+) and MDA-MB-231^WT^ (ER*α*−) cells at different ratios and MCF-7 alone group. In the 100% ER*α*+/ER*α*− ratio group, ER*α* protein expression was as high as observed in MCF-7 cells. With decreasing ER*α*+/ER*α*− ratio, the expression of ER*α* protein also decreased gradually. At the 0% ER*α*+/ER*α*−ratio group, ER*α* protein did not express at all. (b) Analysis of ER*α* gene expression by RT-PCR at different ER*α*+/ER*α*− ratio groups in tumor tissue. ER*α* expression decreased proportionally with decrease in the ER*α*+/ER*α*−ratio.

**Figure 3:** Invasion and migration assay *in vitro*. (a) 1/2: The numbers of cells that crossed the Matrigel filter showed that cell invasion ability significantly stabilized at 40% and 70% ER*α*+/ER*α*−ratio. (b) 1/2: Compared to the MCF-7 group (control), in the 70% ER*α*+/ER*α*− ratio group, the most cells migrated rapidly and scratches became significantly narrow after 24h; after 48 h, the scratches were completely filled with cells.

The article "Role of Estrogen Receptor-Positive/Negative Ratios in Regulating Breast Cancer" was published in 2022. Journal: Evid Based Complement Alternat Med.

**Figure 4:** TNF-*α* and VEGF expression analysis in tumor tissue by immunohistochemical assay. TNF-*α* and VEGF expression were strongly positive (+++) in 40% and 70% ER*α*+/ER*α*− ratio groups, compared to 20% and 0% ratio groups (*P* < 0.05). No staining or number of positively stained cells <10% was considered as negative staining; Light yellow and positively stained cells <11% ≤ 25% were weakly positive (+). Brownish yellow and 26% < positively stained cell ≤50% were medium positive (++); positively stained cells ≤51% was strongly positive (+++).

**Figure 5:** The ER*α*+/ER*α*− ratio plays a critical role in the tumor microenvironment. (a) 1/2: M2 type macrophage polarization at different ER expression levels in tumor microenvironment. M2 macrophage polarization was induced significantly (*P* < 0.05) in the 70% ER*α*+/ER*α*− ratio group. (b) BRCA1 and HER-2 expressing in tumor tissue. BRCA1 and HER-2 expression were induced significantly (*P* < 0.05) in 40% and 70% ER*α*+/ER*α*− ratio groups.

## Data Availability

No data were used to support this study.
